# Influence of Standardized Nursing Management of Hospital Based on Smart Electronic Medical Blockchain on Nursing Quality of Digestive Endoscopy Room

This article has been retracted.

**DOI:** 10.1155/2021/5539901

**Published:** 2021-04-26

**Authors:** Yufen Niu

**Affiliations:** Inner Mirror Room, Zhangqiu District Hospital of Traditional Chinese Medicine, Zhangqiu 250200, Jinan, China

## Abstract

With the increase of the incidence rate of digestive system diseases, digestive endoscopy has become an essential measure. The nursing quality of digestive endoscopy room will have a direct impact on the examination results and treatment effect, so improving the nursing quality of digestive endoscopy room has always been the focus of attention. In this paper, the smart electronic medical blockchain technology and hospital standardized nursing management mode are combined to develop the smart medical standardized nursing management mode. Firstly, 88 patients with digestive endoscopy in a hospital from October 2018 to October 2019 were selected as the experimental subjects: 44 cases in the control group and 44 cases in the experimental group. The control group implemented the traditional management mode of digestive endoscopy room, and the experimental group implemented the standardized nursing management mode of smart medicine. The blood pressure level before and after nursing and the probability of adverse reactions in the process of nursing were counted. After nursing, the patients were asked to fill in the nursing satisfaction questionnaire, evaluate the nursing quality of nursing staff, and make statistics and comparison on the occurrence of safety events in digestive endoscopy room. After nursing, the systolic pressure drop of the experimental group was 125.36 ± 7.27 mmhg, diastolic pressure drop was 73.24 ± 4.21 mmhg, and the incidence of adverse reactions was 11.36%. The satisfaction rate of the experimental group was 15%, 29.55%, and 22.73% higher than that of the control group. The average scores of nursing skills, operation level, and examination results of nursing staff in the experimental group were 94.49, 95.12, and 95.89, respectively; the qualified rate of disinfection of digestive endoscopy room in the experimental group was 100%, the degree of cooperation between doctors and nurses was 100%, the timely rate of emergency measures was 95.45%, and the incidence of accidents was 0%. This shows that, under the standardized nursing of smart medicine, the blood pressure of patients is more stable, the incidence of adverse reactions is lower, the nursing satisfaction is higher, and the nursing quality of nursing staff and the safety of digestive endoscopy room are also improved.

## 1. Introduction

### 1.1. Background Significance

Digestive endoscopy is widely used in the diagnosis and treatment of digestive system diseases. Because the examination is an invasive operation, patients will inevitably have discomfort [1]. The quality of nursing work in digestive endoscopy room will directly affect the treatment effect and also affect the management quality and social image of the hospital. Therefore, it is an urgent problem to improve the quality of nursing and the medical experience of patients in digestive endoscopy room. Smart e-health applies information and computer technology to the medical system, providing convenient smart medical services for patients and medical institutions [2, 3]. Therefore, this paper studies the nursing management of digestive endoscopy room based on smart electronic medicine and block chain technology, which can provide more data support for the popularization of smart medicine in digestive endoscopy room.

### 1.2. Related Work

Intelligent medicine applies artificial intelligence algorithm to the medical field [4], which brings about great convenience to the daily work and management of the medical field. FP-growth algorithm is an association rule algorithm that does not produce candidate set. It has high practical value in the face of the rapid growth of data volume in intelligent medical system. Because FP-growth is a memory resident algorithm, when it is used in large data sets, it will be powerless. Xu F. combines Hadoop with FP-growth algorithm and compares the performance of single machine and distributed environments through the actual analysis of traditional Chinese medicine data [5]. Deep reinforcement learning combines deep learning model with reinforcement learning algorithm and has achieved great success in computer games, robots, and other fields [6]. In particular, it combines deep reinforcement learning with medical big data generated and collected by medical Internet of things [7]. Liu Z. focused on the potential of deep reinforcement learning in lung cancer detection and proposed several representative deep reinforcement learning models, which may be used in lung cancer detection [8]. In addition, he summarized the common types of lung cancer and the main characteristics of each type.

In order to realize the benefits of personalized medicine, it is necessary to expand the scope of genome testing and consulting. Davison N. aims to evaluate the feasibility of a standardized gene therapy model for inherited retinal dystrophy (IRD) and quantify its impact on patients using selected measures [9, 10]. He recruited 98 patients affected by IRD to receive standardized multidisciplinary care and used checklists to assess the fidelity of the care process. Patients cannot wear masks, so the risk of exposure to COVID-19 is higher. Digestive endoscopy room is a relatively high-risk area of COVID-19 infection. On this basis, Xiao-Peng, combining relevant policies and regulations, formulated the prevention and treatment plan of COVID-19 pneumonia in digestive endoscopy room, in order to prevent hospital infection of COVID-19 [11]. Their research results are conducive to the improvement of nursing quality in digestive endoscopy room, but they do not explain the influence of hospital standardized management on nursing quality in digestive endoscopy room from a systematic perspective.

### 1.3. Innovative Points in This Paper

In order to improve the nursing quality of digestive endoscopy room, create a good medical environment for patients, and improve comfort, this paper analyzes the nursing quality of digestive endoscopy room under standardized nursing management based on smart medical blockchain technology. The innovations of this paper are as follows: (1) The intelligent electronic medical block chain technology is combined with the hospital standardized nursing management mode, and the standardized nursing management mode of the intelligent medical is developed. (2) Comparing the nursing quality of the traditional management mode and the standardized nursing management mode of smart medicine, the experimental results show that the standardized nursing management mode of smart medicine can significantly improve the nursing quality of digestive endoscopy room.

## 2. Smart Electronic Medical Blockchain and Hospital Standardized Nursing Management

### 2.1. Smart Electronic Medical Technology

#### 2.1.1. Smart Medical Service Design

Service design needs to be people-oriented, with the needs of users as the standard to measure the content and way of services provided. The goal of smart medical service design is to make the patient's medical treatment become a more convenient and fast thing and make the hospital's service more efficient and safe [12].

The elements of service design mainly include user value, service, and contact point [13, 14]. The identity of patients in the service design is the user [15], so they become the main receiver and face of the service. Service can be divided into two levels: basic service to solve basic needs and personalized service to solve special needs [16]. Touch point is the key to optimize and improve the service experience. Contact points can be divided into three types: physical level, digital level, and emotional level.

In order to design the service, we should first introduce the theme and design the framework, then brainstorm and state the theme, and determine the specific research plan according to the theme. Then, we conduct field investigation, experience the real situation, and optimize the design pertinently. The third step is to create and find the market positioning through competitive product analysis and create a set of improved service designs according to the research results. The fourth step is to synthesize all the designs, form a user itinerary diagram, describe the existing services, and plan the future services. Finally, the design scheme is communicated to the users to obtain the feedback results, and the service design is continuously improved according to the feedback. The system architecture of smart medicine is shown in Figure 1.

#### 2.1.2. Cloud Service Model

Smart medical cloud service model can be dynamically scalable [17]. Elastic scaling can increase or decrease the usage of computing resources according to the load of services. Vertical scaling can increase memory, but it cannot guarantee the continuity of services. Horizontal scaling can enhance the computing power by changing the number of servers to ensure the continuity of services. Therefore, the elastic scaling model commonly used in cloud service model is horizontal scaling [18].

Elastic scaling algorithms include reactive scaling algorithm and predictive scaling algorithm [19]. When some performance parameters of the system reach the critical conditions, the reactive algorithm will respond and readjust the computing resources. The algorithm has high dependence on the threshold set by users [20]. If the threshold is not set properly, it will have a negative impact on the accuracy of the algorithm. Moreover, the reactive algorithm has a certain lag when it reflects the current load state of the system.

Predictive scaling algorithm can calculate the number of scaling resources according to the predicted value and predict the load in advance. The general formula of moving average prediction algorithm (MA) is shown in the following formula:

(1) $$\begin{array}{c} \text{SMA}=e_{1}x_{t}+e_{2}x_{t-1}+e_{3}x_{t-2}+\cdots +e_{m}x_{1}, \end{array}$$

where *m* is the discrete time point and *e*_1_, *e*_2_,…, *e*_*m*_ is the weight of each time point. The formulas of weighted moving average and exponential moving smoothing are shown as follows:

(2) $$\begin{array}{c} \text{WMA}=\frac{\sum_{i=1}^{m}ix_{i}}{\sum_{i=1}^{m}i}, \end{array}$$

(3) $$\begin{array}{c} \text{EMA}=\varpi x_{t}+\varpi \left(1-\varpi \right)x_{t-1}+{\left(1-\varpi \right)}^{2}x_{t-2}+\cdots +{\left(1-\varpi \right)}^{m-1}x_{t-m+1}, \end{array}$$

where *ϖ* is the smoothing factor, and its value is generally shown in the following formula:

(4) $$\begin{array}{c} \varpi =\frac{2}{m+1}, \end{array}$$

The mathematical expressions of AR and ARMA are shown in the two following formulas, respectively:

(5) $$\begin{array}{c} X_{t}=s+{\sum_{i=1}^{j}\delta }_{i}X_{t-i}+\theta_{t}, \end{array}$$

(6) $$\begin{array}{c} X_{t}=s+\theta_{t}+\sum_{i=1}^{j}\delta X_{t-1}+\sum_{k=0}^{j}\vartheta_{k}\theta_{t-k}, \end{array}$$

where *s* is a constant term, which can be ignored. The input parameter performance matrix of the multi-index prediction model is as follows:

(7) $$\begin{array}{c} D=\left[\begin{array}{cccc} x_{11} & x_{12} & \ldots & x_{1a}\\ x_{21} & x_{22} & \ldots & x_{2a}\\ \vdots & \vdots & \vdots & \vdots \\ x_{b1} & x_{b2} & \ldots & x_{ba} \end{array}\right]. \end{array}$$

The matrix is transformed into a vector, which contains the predicted values of each performance parameter. According to the vector, the weighted moving average formula is used to calculate the expansion index, as shown in the following formula:

(8) $$\begin{array}{c} S=\frac{\sum_{s=1}^{m}sp_{s}}{\sum_{s}^{m}s}. \end{array}$$

#### 2.1.3. Artificial Intelligence Technology

In the intelligent medical system, data mining technology is essential [21, 22]. The accuracy and applicability of association rule analysis are generally expressed by confidence and support, as shown in the two following formulas:

(9) $$\begin{array}{c} \text{confidence}=\frac{\left|\left\{T:X\cup Y\subseteq T,T\in Q\right\}\right|}{\left|\left\{T:X\subseteq T,T\in Q\right\}\right|}100\%, \end{array}$$

(10) $$\begin{array}{c} \sup\text{pport}=\frac{\left|\left\{T:X\cup Y\subseteq T,T\in Q\right\}\right|}{\left|Q\right|}100\%. \end{array}$$

The most simple and common classification algorithm is k-nearest neighbor algorithm, and its decision rules in the training set are shown in the following formula:

(11) $$\begin{array}{c} P\;\left({\bar{c}}_{t},d_{j}\right)=\sum_{u_{j}\in \text{KNN}}\text{sim}\left({\bar{c}}_{t},{\bar{u}}_{j}\right)y\left({\bar{u}}_{j},d_{j}\right)-a. \end{array}$$

The similarity between the test text vector and the training text vector is as follows:

(12) $$\begin{array}{c} \text{sim }\left({\bar{c}}_{t},{\bar{u}}_{j}\right)=\frac{\sum_{k=1}^{v}w_{tk}\times w_{jk}}{\sqrt{\sum_{k=1}^{v}{\left(w_{tk}\right)}^{2}}\sqrt{\sum_{k=1}^{v}{\left(w_{jk}\right)}^{2}}}. \end{array}$$

The entropy required by the sample of decision tree theory is shown in the following formula:

(13) $$\begin{array}{c} E\left(t_{1},t_{2},\ldots ,t_{m}\right)=-\sum_{i=1}^{m}p_{i}\log_{2}\left(p_{i}\right), \end{array}$$

where *t* is the number of samples. The entropy of *T* data sample set divided by noncategory attribute *F* is shown in the following formula:

(14) $$\begin{array}{c} E\left(F\right)=-\sum_{j=1}^{v}\frac{t_{1j}+\cdots +t_{mj}}{T}E\;\left(t_{ij},\ldots ,t_{mj}\right). \end{array}$$

The information gain ratio is shown in the three following formulas:

(15) $$\begin{array}{c} GR\left(F,T\right)=\frac{G\left(F,T\right)}{SI\left(F,T\right)}, \end{array}$$

(16) $$\begin{array}{c} G\left(F,T\right)=E\left(t_{1},t_{2},\ldots ,t_{m}\right)-E\left(F\right), \end{array}$$

(17) $$\begin{array}{c} SI\left(F,T\right)=-\sum_{i=1}^{c}\frac{\left|T_{i}\right|}{\left|T\right|}\log_{2}\frac{\left|T_{i}\right|}{\left|T\right|}, \end{array}$$

### 2.2. Blockchain Technology

#### 2.2.1. Level of Blockchain

Blockchain is a decentralized distributed database maintained collectively. In order to prevent data from being tampered, it also uses cryptography to store data. The data layer of blockchain technology is responsible for recording information, which is mainly composed of data blocks recording data information, chain structure containing block main chain, time stamp arranged in chronological order, hash function of mapping data, Merkle tree, and nonheap encryption algorithm [23, 24]. The node uses the hash function and the Merkle tree to store the content received in one cycle in a block, which can be added to the blockchain once the block is approved [25].

The network layer of blockchain can let all nodes in the network maintain the content and effectiveness of the block together in a decentralized structure. The network layer includes peer-to-peer network propagation mechanism and verification mechanism. Peer-to-peer network realizes decentralization by changing the server centric situation, and it can also discard invalid information in a certain period of time to avoid some malicious attacks [26]. The dissemination mechanism ensures that effective information is disseminated throughout the network and proof of workload is found [27]. The verification mechanism can detect whether the data in the block is valid and add the valid information to the main blockchain.

The formula layer of the blockchain can make the distrusted nodes with decentralized decision-making power reach a consensus in the case of decentralization. POW mechanism ensures the security of consensus based on workload proof [28]. POS mechanism is proof of equity, and the rights and interests of different nodes will be different. DPoS mechanism is to appoint the certificate of equity and elect some representative nodes to be responsible for the consensus process of the block. If the elected node has problems, other nodes can work instead of it [29].

#### 2.2.2. Technical Features of Blockchain

Blockchain has the characteristic of being distributed, and the encrypted data is stored in the terminal devices [30]. Blockchain also has the characteristic of collective maintenance, and all nodes with maintenance function can participate in the maintenance work.

Blockchain has the characteristic of decentralization. There is no centralized hardware or management organization in the network, and all nodes are equal to each other. The calculation failure or loss of a single node will not affect the operation of the whole system [31]. Blockchain also has the characteristic of trust, which realizes the transparency of system data operation and the disclosure of data content through the way of distributed account books [32]. Even if there is no mutual information between data, transactions can be carried out.

Blockchain is a reliable database, which cannot modify a single node. Its security is fully guaranteed, and its authenticity is more reliable. Blockchain also has the characteristics of programmability and expandability [33], and intelligent contract does not need too much intervention.

#### 2.2.3. Problems of Blockchain Technology

Blockchain technology is still in the stage of research and development, so there are some problems. Firstly, the data writing speed of blockchain is slow, the period of modification and update is long, and the update of transaction data will lag, which will reduce the overall efficiency [34]. Then there is the problem of energy consumption. The computing engineering of blockchain is huge, and the corresponding energy consumption is also great [35], which will have a great impact on resources and environment.

There are still some potential security risks in the application of blockchain, mainly some malicious attacks from the Internet. The node information of blockchain is huge, and once attacked, the consequences are unimaginable. In addition, blockchain technology has “Mundell Impossible Triangle” [36]. The efficiency and energy consumption of public chain are low, and it has high fairness, but it is not suitable for commercial use. The fairness of the alliance chain is general, and the efficiency will be improved with the improvement of energy consumption [37].

There is a game problem in blockchain [38]. In some unregulated corners, the profit driven market will lead to the use of blockchain in illegal fields. Technological innovation based on blockchain will bring about local or regional financial risks, which may violate the financial law [39], because only relying on technological progress cannot guarantee the orderly operation of finance.

### 2.3. Hospital Standardized Nursing Management

#### 2.3.1. Nursing Management Methods

Nursing management is a key link in hospital nursing. The quality of this link has a great impact on patients' satisfaction and comfort. At present, the commonly used nursing management methods are 5S management method and 6S management method [40, 41]. 6S management method adds “SECURITY” to 5S management method. In the management of hospital nursing [42], the specific management mode of 6S management method is as follows.

The first is “SEIRI,” which divides all medical devices and drugs in hospital nursing workplace into necessary and unnecessary and only leaves the necessary ones to prevent misuse and expand the usable space. The second is “SEITON.” The necessary items left in the previous step should be placed in order and marked to shorten the search time. The third is “SEISO,” which is to standardize the placement and management of all items in the studio, so as to reduce the damage to medical devices [6]. The fourth is “SEIKETSU,” which is mainly used to maintain the results of the above steps. The fifth is “SHITSUKE,” where nursing staff should develop good habits, carry out nursing work according to the rules, and create team spirit. The sixth is “SECURITY,” which needs to establish a safe nursing environment.

All links of 6S management method are connected with each other and complement each other. We need to follow the implementation principles of efficiency, humanization, and aesthetics [43]. Since the implementation of 6S management method in the field of hospital nursing, it has brought about many benefits. 6S management creates a clean and tidy environment and improves the image of the hospital. It can increase the service life of medical devices, reduce the waste of medical supplies and drugs, and reduce the management cost [44].

#### 2.3.2. Standardization Index

Standardization of nursing work: when carrying out nursing work, medical staff need to work in strict accordance with the process and rules and regulations; check the number of medical items every day and timely check whether there are potential safety hazards in medical devices [45]; formulate emergency treatment measures for accidents; and assess the nursing work of various departments, hold regular meetings, and timely analyze and correct problems.

Standardization of medical documents: patients should read all kinds of medical documents before operation, have a certain understanding of the risks of their upcoming operation or examination, and let them sign after obtaining the understanding and consent of patients; nursing medical records must also be written in accordance with relevant regulations and norms [46].

Environmental maintenance standardization: the environment of the nursing room should be standardized, and standardized standards should be formulated for the placement and check of items, such as classified placement and regular check by special personnel; besides remaining clean and tidy, the nursing room must also be equipped with commonly used consumable nursing supplies to meet the daily needs, provide patients with a full range of nursing services, and improve the quality of the environment.

## 3. Nursing Experiment in Digestive Endoscopy Room

### 3.1. Clinical Data and Methods

88 patients with digestive endoscopy in a hospital from October 2018 to October 2019 were selected as the experimental subjects and randomly divided into the control group and the experimental group with 44 cases in each group. The control group was given the number 0, and the experimental group was given the number 1.

The control group implemented the traditional management mode of digestive endoscopy room and arranged the daily nursing work reasonably. The experimental group implemented the standardized nursing management mode based on intelligent medical treatment. The research roadmap of this paper is shown in Figure 2.

### 3.2. Standardized Nursing Management Mode Based on Smart Medicine

Set up standardized nursing team, and train the team members on the use of smart medical technology.

The digestive endoscopy room needs to maintain appropriate temperature and humidity, ensure that there is half an hour of ventilation time every day, and conduct an hour of ultraviolet disinfection.

Put the articles in the digestive endoscopy room reasonably, and use the intelligent medical system to know the inventory and use of drugs in time.

Eliminate the bad mood of patients before digestive endoscopy examination, and pay attention to the feelings of patients in time during the examination. If there are adverse reactions, they should be appeased and treated in time.

In the process of diagnosis and nursing, the information and treatment of patients will be timely filled in the electronic medical records and files, and the data will be processed, comprehensively understanding the patient's condition to ensure the quality of care.

### 3.3. Observation Indexes

Before nursing, the general data of patients were counted, including age, gender, and course of disease distribution. The blood pressure levels of the two groups before and after nursing were counted, and the occurrence of adverse reactions in the nursing process was recorded.

After the nursing, the patients were asked to fill in the nursing satisfaction questionnaire, including the satisfaction survey on the environment, work efficiency, and nursing attitude of the endoscopy room. The satisfaction rate is the ratio between the number of people who are very satisfied and generally satisfied and the total number of people.

Evaluate the nursing quality of nursing staff, mainly including nursing technology, operation level, and examination results. The occurrences of safety incidents in digestive endoscopy room were counted and compared, mainly including qualified disinfection, reasonable medical cooperation, timely first-aid measures, and accidents.

## 4. Discussion on Nursing Quality of Digestive Endoscopy Room

### 4.1. Incidence of Adverse Reactions

#### 4.1.1. General Information of Patients before Nursing

According to the information in the electronic medical records, the distribution of age, gender, and course of disease (month) of the two groups was as follows.

As shown in Table 1, the male-to-female ratio in the control group was 24 : 20, the mean age was 47.4 ± 4.8 years, and the course of disease was 3–23 months. The male-to-female ratio in the experimental group was 23 : 21, the mean age was 51.1 ± 5.2 years, and the course of disease was 3–28 months. The data showed that the two groups were comparable in terms of gender, age, and course of disease.

#### 4.1.2. Changes of Blood Pressure before and after Nursing

The blood pressure levels of patients before and after nursing were detected and compared.

As shown in Figure 3, after nursing, the systolic blood pressure of the experimental group decreased from 147.34 ± 15.21 mmHg to 125.36 ± 7.27 mmHg, and the diastolic blood pressure decreased from 85.57 ± 9.11 mmHg to 73.24 ± 4.21 mmHg. In the control group, systolic blood pressure decreased from 147.52 ± 16.34 mmHg to 125.36 ± 11.39 mmHg, and diastolic blood pressure decreased from 85.37 ± 9.39 mmHg to 76.15 ± 5.14 mmHg. This shows that, under the standardized care of smart medicine, the psychological mood of patients has been relieved to a certain extent, and the blood pressure is more stable.

#### 4.1.3. Incidence of Adverse Reactions in Nursing

In the nursing process, two groups of patients with cough, vomiting, and physical discomfort of adverse reactions were statistically analyzed.

As shown in Table 2, the total number of patients with adverse reactions in the experimental group was 5, and the total incidence of adverse reactions was 11.36%. The total number of adverse reactions in the control group was 13, and the total incidence of adverse reactions was 29.55%.

As shown in Figure 4, in the experimental group, there were 2 cases of cough, 1 case of vomiting, and 2 cases of physical discomfort, and the cumulative number of adverse reactions was 5; in the control group, there were 3 cases of cough, 4 cases of vomiting, and 6 cases of physical discomfort, and the cumulative number of adverse reactions was 13. The incidences of adverse reactions were calculated and compared.

As shown in Figure 5, in the experimental group, the probabilities of cough, vomiting, and physical discomfort were 4.55%, 2.27%, and 4.55%, respectively, and the total incidence of adverse reactions was 11.36%. In the control group, the probabilities of cough, vomiting, and physical discomfort were 6.82%, 9.09%, and 13.64%, respectively, and the total incidence of adverse reactions was 29.55%. This shows that, under the standardized care of smart medicine, the probability of adverse reactions of patients undergoing digestive endoscopy is lower, and the comfort is higher.

### 4.2. Patient Care Satisfaction

#### 4.2.1. Satisfaction of Patients in the Control Group

The patients in the control group were satisfied with the environment, work efficiency, and nursing attitude of the endoscopy room.

As shown in Figure 6, 24, 21, and 22 patients in the control group were very satisfied with the environment, work efficiency, and nursing attitude of the endoscopy room; 13, 17, and 15 patients were dissatisfied; the satisfaction rates were 70.45%, 61.36%, and 65.91%, respectively. This shows that the patients in the control group under the traditional management mode of digestive endoscopy room are not satisfied with the nursing.

#### 4.2.2. Satisfaction of Patients in the Experimental Group

The satisfaction of patients in the experimental group with the environment, work efficiency, and nursing attitude of the endoscopy room was as follows.

As shown in Figure 7, 33, 30, and 29 patients in the experimental group were very satisfied with the environment, work efficiency, and nursing attitude of the endoscopic room; 2, 4, and 5 patients were dissatisfied; the satisfaction rates were 95.45%, 90.91%, and 88.64%, respectively. This shows that the experimental group based on the standardized nursing management mode of smart medicine has a higher satisfaction rate of nursing.

#### 4.2.3. Comparison of Satisfaction Rate between the Two Groups

The two groups of patients were summarized and compared in terms of the endoscopic room environment, work efficiency, and nursing attitude satisfaction data.

As shown in Table 3, the satisfaction rate of the experimental group was 15% higher than that of the control group, 29.55% higher than that of the control group, and 22.73% higher than that of the medical staff. This shows that the patient satisfaction of standardized nursing management mode based on smart medicine is higher than that of traditional nursing mode.

### 4.3. Nursing Quality Evaluation

#### 4.3.1. Nursing Quality of Nursing Staff

The nursing quality of 6 nurses in the experimental group and the control group was evaluated randomly. The number of nurses in the experimental group was E1–E3, and the number of nurses in the control group was C1–C3. The full score was 100. The higher the score, the higher the quality.

As shown in Figure 8, the scores of nursing technique, operation level, and examination result of the nursing staff in the experimental group were 94.49, 95.12, and 95.89, respectively. The scores of nursing technique, operation level, and examination results of the nursing staff in the control group were 77.07, 78.83, and 78.63, respectively. The scores of the two groups were significantly different. This shows that the nursing quality of the experimental group is higher than that of the control group. The combination of intelligent medicine and standard management is conducive to improve the nursing technology, operation level, and examination results of the medical staff.

#### 4.3.2. Safety and Quality of Digestive Endoscopy Room

The occurrences of safety incidents in digestive endoscopy room were counted and compared, mainly including qualified disinfection, medical cooperation, timely emergency measures, and accidents.

As shown in Figure 9, the qualified rate of disinfection in the digestive endoscopy room of the experimental group was 100%, the degree of cooperation between doctors and nurses was 100%, the timely rate of emergency measures was 95.45%, and the incidence of accidents was 0%. In the control group, the qualified rate of disinfection was 79.54%, the degree of cooperation between doctors and nurses was 75%, the timely rate of emergency measures was 77.27%, and the incidence of accidents was 11.36%. This shows that the standardized nursing management mode of smart medicine is helpful to reduce the incidence of safety incidents in digestive endoscopy room.

## 5. Conclusions

Digestive endoscopy is widely used in the diagnosis and treatment of digestive system diseases. As the examination is an invasive procedure, patients will inevitably have discomfort. In severe cases, patients will refuse to check, so the quality of nursing work in digestive endoscopy room will directly affect the treatment effect and also affect the management quality and social image of the hospital. Therefore, it is urgent to improve the quality of nursing in digestive endoscopy room and the medical experience of patients.

In this paper, the smart electronic medical blockchain technology and hospital standardized nursing management mode are combined to develop a smart medical standardized nursing management mode for digestive endoscopy room nursing. First of all, a standardized nursing team was set up to maintain the appropriate temperature and humidity in the digestive endoscopy room, ventilation, and disinfection on time. Put the articles in the digestive endoscopy room reasonably and use the drug management system of smart medicine to understand the inventory and use of drugs in time. Eliminate the bad mood of patients before digestive endoscopy examination, and pay attention to the feelings of patients in time during the examination. If there are adverse reactions, they should be appeased and treated in time. In the process of diagnosis and nursing, the information and treatment of patients will be timely filled in the electronic medical records and files, and the data will be processed, comprehensively understanding the patient's condition to ensure the quality of care.

The objective was to compare the nursing quality between the traditional management mode of digestive endoscopy room and the standardized nursing management mode of smart medicine. The experimental results showed that, under the standardized nursing of intelligent medical care, patients' blood pressure was more stable, the incidence of adverse reactions in the nursing process was lower, and the satisfaction of nursing was higher. The quality of nursing work and the safety quality of digestive endoscopy room have also been improved.

## Figures and Tables

**Figure 1:** System architecture of smart medicine.

**Figure 2:** Research roadmap.

**Figure 3:** Changes of blood pressure before and after nursing.

**Figure 4:** Incidence of adverse reactions.

**Figure 5:** Incidence of adverse reactions.

**Figure 6:** Satisfaction of patients in the control group.

**Figure 7:** Patients' satisfaction in the experimental group.

**Figure 8:** Nursing quality score of nursing staff.

**Figure 9:** Incidence of safety events in digestive endoscopy room.

**Table 1:** General information of patients.

Group	Average age	Male	Female	Course of disease (months)
Experience group	47.4 ± 4.8	24	20	3∼23
Control group	51.1 ± 5.2	23	21	3∼28

**Table 2:** Incidence of adverse reactions in two groups.

Adverse reactions		Experience group	Control group
Choking cough	Number of cases	2	3
	Incidence rate	4.55%	6.82%
Vomit	Number of cases	1	4
	Incidence rate	2.27%	9.09%
Malaise	Number of cases	2	6
	Incidence rate	4.55%	13.64%

**Table 3:** Comparison of nursing satisfaction.

Group	Environment (%)	Efficiency (%)	Attitude (%)
Experience group	95.45	90.91	88.64
Control group	70.45	61.36	65.91
Difference	15	29.55	22.73

## Data Availability

No data were used to support this study.
